This article has been retracted.

# Effect of Core Strength Training on Rehabilitation of Chronic Low Back Pain in Aerobics Athletes

**DOI:** 10.1155/2022/8740665

**Published:** 2022-05-09

**Authors:** Xi He

**Affiliations:** College of Physical Education, Qilu Normal College, Jinan 250013, Shandong, China

## Abstract

Chronic low back pain, as a common disease of aerobics athletes, has caused a lot of problems for aerobics athletes, and core strength training can form a strong back muscle through the back muscle training to maintain support functions. Maximize the physiological function of the spine to achieve the effect of treating chronic low back pain. To this end, this article raises the effect of core strength training on the chronic low back pain of aerobics athletes. This article uses electric traction as a control and conducts research by setting up a control experiment. Clinically, the ODI questionnaire is a commonly used judgment criterion for the diagnosis of lumbar function. This article uses the ODI questionnaire as the judgment criterion. The research in this article found that after the experiment, the subjects with a significant decrease in the ODI questionnaire scores in the two groups in the three surveys after treatment were over 80% of the total number in each group, indicating that core strength training is the same as traction therapy. In terms of the effect of treating chronic low back pain, it has obvious effects, and the method in this article is significantly better.

## 1. Introduction

Chronic low back pain refers to a small pain in the back and lumbosacral region, with or without radiation pain in the lower extremities, with a course of more than 3 months. About two-thirds of adults have suffered from low back pain during their lifetime, especially chronic low back pain, which has a long delay and is difficult to obtain accurate diagnosis and appropriate treatment. Therefore, this study will focus on this aspect of chronic low back pain.

With the development of competitive sports and the popularization of aerobics, aerobics has become a common sport at present. Many colleges and universities have launched aerobics courses, and aerobics has gradually gained a place in competitive sports. Chronic low back pain is a common disease among aerobics athletes. It afflicts most aerobics athletes. At present, the treatment of chronic low back pain is still in the exploratory stage. There is no perfect treatment. Core strength training is a proactive therapy. It has an important role in improving the waist function and quality of life of patients. Therefore, it is of great significance to study the effect of core strength training on aerobic athletes' chronic low back pain.

Shmagel explores the effects of intensive physical core strength training on the trunk and knee extensors in patients with chronic low back pain. Shmagel selected 30 patients with chronic low back pain as the research subjects, took their multifidus and lateral femoral muscles for biopsy, measured the size of type 1 and type 2 muscle fibers, and measured isokinetic trunk and knee extensions at two different angular velocities. Anna Shmagel's results showed that the volume of type 2 muscle fibers in male multifidus increased by 11% (*P* < 0.05), and the volume of type 2 muscle fibers in lateral femoral muscle increased by 8% (*P* < 0.05). The corresponding increase in women was 11% (*P* = 0.16) and 11% (*P* < 0.05). The correlation between the size of type 2 muscle fibers in the multifidus muscles and the strength of trunk extension improved, especially in men during the follow-up period. Shmagel's research results show that training with maximum or submaximum strength can reverse the selective atrophy of male multifidus type 2 fibers, and intensive training can also significantly increase the trunk extension strength of women, but women may need longer training time than men to achieve significant structural changes in the back muscles [1]. In order to explore the effect of active rehabilitation on the functional ability and quality of life of patients with chronic low back pain, Bramoweth selected 13 patients with chronic low back pain using a back-and-forth measurement method, and randomly divided them into experimental and control groups of 15 cases each. The experimental group was treated with active rehabilitation 10–30 times, 30 minutes each time. Bramoweth's research results show that active rehabilitation has significant effects on improving physical activity, quality of life, and cognitive behavioral strategies, indicating that active rehabilitation treatment has a significant effect on improving the functional capacity and quality of life of patients with chronic low back pain [2]. Coulombe explores the effects of a new enhanced core stability training technique on physical function, pain, and core stability in patients with chronic low back pain. Coulombe selected 40 patients with low back pain and divided them into two groups for randomized controlled trials. The experimental group was organized except for abdominal wall traction and ankle dorsiflexion; the control group only had abdominal wall traction, and both groups received the same conventional physical therapy training, 3 days a week for 8 consecutive weeks. Brian J Coulombe's experimental results showed that the experimental group had a significant improvement over the control group 2 months after the intervention. Coulombe's research results provided a clinical basis for patients with chronic low back pain who add ankle dorsiflexion to abdominal wall traction, and improved the efficacy in terms of limb disability, pain, and core stability [3].

Aerobics is a kind of physical fitness exercise. Chronic low back pain is a common disease of aerobics athletes. In this article, the effect of core strength training on the chronic low back pain of aerobics athletes was studied. This article first introduced the aerobics exercise, explained the chronic low back pain, and set up a control experiment to compare the effects of core strength training and electric traction on chronic low back pain.

## 2. Proposed Method

### 2.1. Aerobics

#### 2.1.1. Origin of Aerobics

Aerobic exercise refers to an exercise method that mainly uses aerobic metabolism to provide the energy required for exercise. Aerobics can be traced back to ancient Greece two thousand years ago. Ancient Greece achieved strong physique and cultivating sentiment by moving rhythmically with music [4]. Later, they gradually discovered that the sport of aerobics can achieve full development by delighting them. In 1999, China officially introduced aerobics rules and monitoring standards. Especially in recent years, China's aerobics sports have continuously created good results in various leagues, and aerobics-related art examinations have also increased year by year. In recent years, aerobics has been formally introduced in school-based courses, and more and more middle schools are exposed to aerobics and love the sport.

#### 2.1.2. Advantages of Aerobics

1. The aerobics exercise has a moderate load, which can improve the body's metabolic energy, improve the function of various nervous systems and organs, enhance physical fitness, and level skills.
2. For the music of aerobics, generally select music with clear points, bright rhythms, and positive movements, which requires a strong tension in the combined movements. In the process, it seeks a sense of balance from the continuously shifting weight, and the intensity of the aerobics exercise can be minimized. It stimulates the excitement of the motor center in the brain layer and increases the energy consumption of the nervous system. During the exercise, due to the characteristics of aerobics, it can pull the joints and muscles of the body's tissues to contract and relax. Slower gymnastics movements, slower rhythms, and aerobics movements lack more energy consumption and the degree of stretching of joints. Therefore, the characteristics of aerobics make it more valuable for exercise.
3. Calisthenics has a variety of fitness effects and to a certain extent, it continuously trains the whole body and mind of the athlete. Let beauty be felt while spreading it and expressing beauty.

#### 2.1.3. Status of Aerobics

Bodybuilding operation is a new sports item. It has developed into a well-known and very distinctive sports item in just 20 years. It has been widely promoted with its unique rhythm, spectacle, and fitness. However, the study of the theoretical significance of aerobics is in a state of stagnation, especially the development and application of aerobics in middle schools, and the culture derived from aerobics is limited by teachers and school culture, and psychological research [5]. In the mid-1980s, the aerobics movement gradually started in the middle school physical education and health curriculum. The adolescents in middle school have developed rapidly in all aspects of their physical fitness and have a strong curiosity and novelty. It has become a popular form of exercise. Modern high school physical education classes are gradually promoting the aerobics as a fresh sport. It can combine volleyball, basketball, and football with a series of arm and step movements and can also be combined with music to strengthen the ability to remember movements. Facing the conflict between physical education curriculum and physical education in physical education classroom, we should always remind ourselves [6, 7]. Physical education serves physical education and develops physical education while preserving the characteristics of physical education. Make students love sports while re-loving sports courses. In order for students to have a positive attitude toward physical education, students must be clear about their needs for physical education. “For the vast majority of students, they have fitness needs, bodybuilding needs, entertainment needs, and self-worth.”

### 2.2. Chronic Low back Pain

#### 2.2.1. Stable Structure of Lumbosacral Region and Chronic Low Back Pain

The spinal lumbosacral segment is the most heavily loaded segment in the human spinal bar. It is colocated with the surrounding stable structure and various connection methods to maintain the stability and flexibility of the spinal lumbosacral segment. Its physiological convexity is suitable for the human body. There are three important roles for sitting, standing, and lying. The lumbosacral vertebrae form a three-joint complex between the lumbar intervertebral disc and the rear facet joints, which is a bony structure that maintains the stability of the lumbosacral vertebra. The ligament stabilization system of the lumbosacral vertebrae is composed of the longitudinal ligament, the posterior longitudinal ligament, the yellow ligament, the superior spinal ligament, the interspinous ligament, and the transverse process ligament. The lumbar muscles that stretch the lumbar spine and the abdominal muscles that flex the lumbar spine constitute the dynamic system of the stable structure of the lumbosacral spine [8].

Some scholars believe that the stability of the lumbosacral vertebrae's stable structure will cause a series of compensatory changes to cause the main pathogenesis of lower back pain. When spinal instability was caused by intervertebral disc degeneration, physiological load can cause excessive deformation of the intervertebral connection. Biomechanical studies have found that there is abnormal activity in the spinal segment with degenerative intervertebral discs, and the load is transferred to the facet joints [9].

Some scholars believe that lower back pain is related to muscle strain, and the back and back muscles stop and contract after fatigue [10] and give the function to the joint ligaments to maintain it so as not to strain it. He used different seating to study the relationship between low back pain and muscles through myoelectric activity beams. When bending down, the back and back muscles were in a flexed position, and the static effects of the head and upper chest made the back muscles and ligaments in a traction-like state—muscle strain.

#### 2.2.2. Anatomical Characteristics of the Lumbar Spine

The lumbar spine is a specialized functional unit of the spine. It is the backbone of the waist tissues. It is connected to the hip joint and is the main part of the trunk. In terms of structure, the lumbar spine is divided into anterior column, middle column, and posterior column. The anterior column is composed of the anterior longitudinal ligament, the vertebra, and the first half of the disc; the middle column is mainly composed of the posterior longitudinal ligament and the posterior half of the disc; the posterior column is mainly composed of the posterior arch, intervertebral nodules, posterior ligaments, and muscles [11]. In terms of function, the range of flexion and extension of the lumbar spine is large. This is because the lumbar intervertebral disc is large, and the vertebral joints have no restrictive effect on the movement. The forms of exercise include flexion, extension, left and right lateral flexion, and rotation. The main tissues that make up the waist are lumbar fascia, muscles, lumbar vertebrae and their connections, and spinal canal tissues. Muscles are the dynamic structure of lumbar vertebra activity. The cooperation of each muscle produces flexion, extension, lateral bending, and rotation. Fascia is a fixing and protecting device for muscles. The lumbar and sacral vertebrae are the parts that bear the most weight on the human body. They transfer the weight of the body above the waist, including stress from back organisms or sports, to the pelvis and lower limbs. Therefore, compared with other vertebrae of the spine, the lumbar spine is the more active part of the human spine. In terms of innervation, according to anatomy, the innervation of lumbar push can be divided into two intervals. The lumbar spine is divided into ventral and dorsal intervals through the coronal plane of the intervertebral foramen. Laterally, the two spaces are separated by the transverse process and the intertransverse process ligament. The ventral space includes the ventral dura mater, intervertebral disc, anterior ligament, and anterior vertebral muscles. The dorsal space includes nerve arches, vertebral joints and ligaments, and internal muscles of the back. The nerve root and the spinal nerve exiting are in between these two intervals, and the nerve conduction and innervation activities are complicated.

#### 2.2.3. Imaging Findings of Chronic Low Back Pain

*(1) Vertebral Body and Disc Changes*. Among the patients with chronic low back pain, the vertebral body and intervertebral discs had the most changes, up to 85.62%. The anterior vertebral bone spurs accounted for 38.11%, the intervertebral space stenosis accounted for 22.25%, and Schmorl nodules accounted for 6.79%. Disc degeneration is reflected by signs of bone spurs, intervertebral space stenosis, and Schmorl nodules. Intervertebral disc degeneration is a physiological law. With the corresponding changes in tissues such as ligaments, muscles, and small joints, the spinal dulium balance is destroyed, and then the body is compensated or decompensated. From the perspective of directly compressing the nerve root, it is generally considered that the anterior vertebral bone spur is of little clinical significance, but the anterior vertebral bone spur can reflect the pathological changes of disc degeneration.

*(2) Facet Joint Changes*. In X-ray and CT manifestations, facet joint changes are manifested in sudden changes in the upper and lower joints, the joint surface is blurred, asymmetry such as a coronal plane, articular surface sclerosis, joint space widening or narrowing, are all degenerative changes sign. When the facet joint degenerates, the intervertebral space gradually narrows. On the one hand, the small joints fixed by the posterior longitudinal ligament and interspinous ligament loosen, and the extensor traction of the vertebra causes the vertebral body to slide backward and compress the nerve, on the other hand, it can strengthen hypertensive arthritis caused by the movement of the small joints compressions of the bone fiber tube. Soft tissue injury can cause dislocation of the facet joint capsule and joint capsule hypertrophy to shrink adjacent intervertebral foramen. The pain in the lower back is transmitted through the posterior primary branches of the L4, 5, and SI.2, 3 nerves, and the reduction of the foramen makes the posterior primary branches necessarily compressed. Therefore, the anatomical changes of lower back pain in the lower back should be worthy of clinical attention.

*(3) Spike Mutation*. Spinous process proliferation becomes sharp, dense, narrow spinous space, and kiss spinous processes are also revealing in functional low back pain. In maintaining the upright position of the spine, the superior spinal ligament, interspinous ligament, yellow ligament, and posterior longitudinal ligament are effective, so the aging of the aforementioned ligaments will inevitably bring corresponding consequences. When the lumbar spine is flexed, the anterior disc pressure increases and the nucleus pulposus is pressed behind, increasing the tension of the fiber annulus and the posterior longitudinal ligament 23. Because the lumbar lordosis and the lumbosacral angle are reduced, the supraspinous ligament, interspinous ligament, yellow ligament, posterior longitudinal ligament, and small joints are in tension-increasing thoughts, and the back muscles are also in tension-like thoughts, causing lower back pain.

*(4) Congenital Mutation*. Congenital lumbosacral deformity is one of the causes of chronic low back pain, and 53.36% of the X-ray data support this view. There are many congenital deformities in the lumbosacral region, which often makes the lumbar strength unbalanced, causes traumatic arthritis, or weakens the attachment of ligaments and muscles. Once adults engage in more physical labor, symptoms can appear. Among them, the recessive spinous process (S1) and the lumbar spine are the most common. Congenital developmental variation, imbalance of activity due to static and dynamic reasons for various reasons, prone to lack and release of small joint ligaments, making the attachment points of the sacrospinalis muscle, superior spinal ligament, and spinal ligament weak or weakening stability, leading to chronic strain. Lumbar vertebralization or sacral vertebralization can cause imbalance of lumbosacral and sacroiliac joints, whether completely or incompletely. Patients with low back pain may have lumbosacral deformities, but those with lumbosacral deformities may not necessarily have low back pain. Therefore, congenital lumbosacral deformities are only a potential internal cause of low back pain.

*(5) Physiological Curvature Change*. The change of lumbosacral dust curvature is an important imaging manifestation in compensatory changes. Among them, the reduction of lumbar anterior arch is the most common. When the spine straightens, the facet joint capsule is tightened, abnormal changes in the upper and lower articular processes occur, and the articular cartilage is compressed. At the same time, the tension of the lumbar and back muscles and fascia is increased, which can make the sacral spine rotate upward and backward. This can increase strain on the sacroiliac joint and its adjacent ligaments and cause strain. Other scoliosis, kyphosis, etc., can also increase the burden on the transverse process ligaments and posterior longitudinal ligaments, the yellow ligaments, and the ligaments of the spinous processes.

#### 2.2.4. Treatment of Low Back Pain

Clinically, the treatment of low back pain is mainly divided into surgical methods and nonsurgical methods. For special groups such as athletes, conservative treatment should be preferred for the treatment of low back pain. In particular, low back pain caused by lumbar muscle injury and ligament strain can usually be restored very well through proper rest and conservative treatment. For waist and leg pain, you can take conservative treatment first, without surgery, commonly used methods, such as applying plaster for promoting blood circulation and removing blood stasis, locally with towel hot compress physiotherapy equipment, baking electricity, acupuncture, moxibustion, pay attention to keep warm, and strengthen rest.

*(1) Effect of Core Strength Training on Chronic Low Back Pain*. Rehabilitation training refers to physical activities that help restore or improve function after an injury. The purpose of core strength training is to promote the healing of injured tissues, correct the mechanical changes of the spine, especially to strengthen the stability of the lumbar spine. In recent decades, people have tended to use functional exercises to systematically improve muscle function to prevent and treat chronic low back pain, a common disease.

*(2) Endurance Training*. Endurance training is aerobic training, which is characterized by low resistance, many repetitions, and long duration, such as walking and jogging. The purpose is to strengthen the function of the cardiovascular system. Aerobic exercise can increase blood flow, reduce peripheral vascular resistance, reduce blood pressure, increase the number of capillaries, mitochondrial density, and oxidase in the metabolic chain, thereby providing sufficient oxygen and nutrients for the activities of the trunk muscles and bones, and promoting elimination of metabolites. Compared with passive physical therapy methods such as hyperthermia and ultrasound, core strength training increases blood perfusion in the affected area by strengthening the role of vascular pump, instead of using external stimuli such as heating, making the effect more secure and reliable. On the other hand, proper exercise can control the patient's weight, improve the patient's psychological function, and reduce pain symptoms.

*(3) Flexibility Exercises*. Flexibility refers to the stretching ability of the joints of the human body, the stretch of muscles and toughness. It mainly depends on the structure of bones, the volume of tissues around the joints, and the stretch elasticity across the ligaments, tendons, muscles, and skin of the joints. Flexibility can be divided into active flexibility and passive flexibility. Active flexibility refers to the range of joint motion that can be achieved by using muscles, while passive flexibility is simply the maximum range of joint motion.

*(4) Traction Treatment*. Traction treatment is currently one of the most commonly used conservative treatments for low back pain. The principle is nothing more than reducing the intervertebral pressure load and alleviating facet joint irritation and back muscle spasm. The key to its treatment is to open the intervertebral space and reduce the pressure load by releasing the intervertebral joints (intervertebral discs and posterior joints).

## 3. Experiments

### 3.1. Experimental Objects and Diagnostic Criteria

#### 3.1.1. Experimental Object

This article selects 60 female athletes from aerobics classes in a college who have suffered chronic low back pain after physical training. After clinical examination in the hospital, the main pathological characteristics of these 60 female athletes are lumbar muscle strain, ligament strain, and no spinal canal—lesions. Sixty athletes were randomly divided into an experimental group (30 people) and a control group (30 people). Traction method is a traditional method for treating low back pain, and its therapeutic effect has been clinically recognized. This article uses traction treatment as a control treatment method to set a control in the experiment; the control group was treated with traction, and the experimental group was treated with core strength training. The age, height, and weight of the two groups were examined. The *P* values were 0.521, 0.802, and 0.522, respectively, and P was greater than 0.05. The difference was not significant. The situation is shown in Table 1.

Table 1 shows that there were no significant differences in age, height, and weight of the subjects.

#### 3.1.2. Diagnostic Criteria

1. Persistent pain between the 12th rib of the lower back and the gluteal groove, with or without posterior lateral femoral radiation pain (not exceeding the knee joint).
2. Complaints of tenderness and/or muscle spasms in and above the pain area.
3. Except for lumbar spine rotation, small joint space narrowing, separation, asymmetry, and other signs on X-ray films, no other positive findings were found on imaging examination.
4. Excluding bone and joint system through laboratory, imaging examination or bone density measurement can cause lower back pain.
5. Exclude other systems that can cause low back pain through laboratory and imaging studies.

#### 3.1.3. Treatment Plan

*(1) Control Group-Electric Traction*. Using a fully automatic lumbar traction machine, remove the hard object from the patient, lie prone on the traction bed, the whole body is in a relaxed state, fix the thorax and pelvis, connect the power supply, and select the appropriate traction force according to the patient's weight and tolerance (usually (half of the patient's weight plus 5–10 kg is the standard), the traction time is 30 min/time, and 2 weeks is a course of treatment. Traction treatment was continued for 2 weeks, a total of 14 times, and the symptoms could be discontinued.

*(2) Experimental Group-Core Strength Training*. Core strength training is carried out according to a simple gymnastic exercise program of strong lumbar and abdominal muscles arranged by professionals. The rehabilitation group is required to train daily for a period of 3 months:

1. Practice frequency: practice once a day, and do two to three groups each time (completion—a set of gymnastic moves is—group).
2. Practice time: about 30 min per practice.
3. Exercise intensity: Try not to increase pain and cause fatigue as much as possible. You can make corresponding adjustments according to the specific conditions of each subject.

### 3.2. Evaluation Index

This article uses the Oswestry Dysfunction Index Questionnaire (ODI). The questionnaire consisted of 10 questions, including the intensity of pain, daily self-care, lifting, walking, sitting, sleeping, social life, and travel. There are six options for each question, and each option is from light to heavy at one time. The first question is 0 points and the last question is 5 points. If all 10 questions are answered, the scoring method is actual score/50 (highest possible score) × 100%, if there is no question answered, the scoring method is: actual score/45 (highest possible score) × 100%. By analogy, the higher the score, the more severe the dysfunction.

This article uses two treatment methods. Although the two methods have different cycles, the evaluation times are the same. They are evaluated once before treatment, at the end of treatment, 2 weeks and 6 weeks after treatment, a total of four times. Patient follow-up, telephone follow-up, or letter follow-up were used to assess patients at the abovementioned time follow-up, and the collected four questionnaire indexes were compared to judge and evaluate the effects of core strength training and electric traction treatment on lower back pain. The ODI questionnaire scores at the end of treatment, 2 weeks after treatment, and 6 weeks after treatment were compared with the scores before treatment, and the decline values were taken. The more the value decreases, the better the treatment effect.

### 3.3. Data Processing

SPSSl5.0 statistical software was used to perform statistical analysis on the measurement data. The results were expressed as mean standard deviation (*M* ± SD). Independent sample *T* test was used to compare the means between groups. Corrected *T* test was used when the variance was uneven.

## 4. Experimental Results and Analysis

### 4.1. Overall Analysis of the Scores of the Four ODI Questionnaires in the Experimental and Control Groups

Within 24 hours before each questionnaire was filled out, all subjects did not perform strenuous physical activity to ensure that the degree of pain reflected in the questionnaire score was close to the true level. The results of the four ODI questionnaire scores in the two groups are shown in Figures 1 and 2.

From the overall analysis of the four ODI questionnaire scores of the experimental group and the control group in Figures 1 and2, it can be seen that after core strength training and traction treatment, the scores of the ODI questionnaire scores after treatment and before treatment show that both groups of subjects have significant improvement in back pain . Among them, for *P* < 0.01 in the rehabilitation group, there was a very significant difference; for *P* < 0.05 in the traction physiotherapy group, there was a significant difference; and the decline in ODI between the two groups showed that the decline in the core strength training group was greater than the control group.

### 4.2. Detailed Comparison of the Scores of the Two Groups of ODI Questionnaires

#### 4.2.1. Changes in the Average SCORE of the Two Groups of ODI Questionnaires

Analysis of the changes in the average score of the two groups of ODI questionnaires, the results are shown in Figure 3.

It can be seen from Figure 3 that after core strength training and electric traction treatment, the ODI scores of both groups of subjects decreased. After 2 and 6 weeks of treatment, the ODI scores showed an increasing trend, but neither exceeded the score before treatment.

#### 4.2.2. Comparison of ODI Questionnaire Scores between the Two Groups

The two groups of ODI questionnaire scores were compared and the results are shown in Figure 4.

It can be seen from Figure 4 that after core strength training and electric traction treatment, the ODI questionnaire scores of the two groups of subjects decreased, indicating that both the physical pain and the disorder index decreased. After 2 and 6 weeks of treatment, the ODI questionnaire scores of returning subjects increased slightly, but they did not exceed the levels before treatment.

#### 4.2.3. Phase Comparison of ODI Questionnaire Scores between the Two Groups

The scores of the ODI questionnaires before and after treatment were compared between the two groups. The results are shown in Table 2.

From the comparison of the ODI questionnaire scores before and after the treatment of the subjects in Table 2, it can be seen that there is a significant difference between *P* < 0.01 and *P* < 0.05.This shows that the treatment is effective, but the effect of the control group is more obvious.

The ODI questionnaire scores of the two groups were compared before treatment and 2 weeks after the treatment. The results are shown in Table 3.

The scores of the ODI questionnaires were compared between the two groups before and 6 weeks after the end of treatment. The results are shown in Table 4.

Tables 3 and 4 show that the scores of the two return visits after the end of treatment in the experimental group are significantly different from the scores of the pretreatment questionnaire (*P* < 0.01), and the control group is significantly different (*P* < 0.05). In addition, the fluctuation of the return visit score 2 weeks after treatment was not as great as the fluctuation of the return visit score after 6 weeks of treatment.

According to Tables 2–4, it can be seen that the ODI questionnaire scores of the experimental group after core strength training for 3 months at the end of treatment, 2 weeks after the end of exercise, and 6 weeks after the end of exercise were significantly different from those before treatment (*P* is less than 0.01). This indicates that core strength training has a positive effect on restoring lumbar function in subjects with chronic low back pain. In addition, the control group received ODI questionnaire scores and treatment after 2 weeks of traction treatment, at the end of treatment, 2 weeks after exercise, and 6 weeks after exercise. There were significant differences in the previous comparisons (all *P* were less than 0.05). This shows that traction treatment can effectively treat chronic low back pain.

#### 4.2.4. Comparison of Scores of ODI Questionnaires between Two Groups

The two groups of ODI questionnaire scores were compared, and the results are shown in Figure 5.

It can be seen from Figure 5 that after the core strength training and electric traction treatment, the subjects with significantly lower ODI questionnaire scores in each group in the three surveys after the treatment end accounted for more than 80% of the total number in each group, indicating core strength training Like traction therapy, it has obvious effects in the treatment of chronic low back pain. As shown in Figure 5, the proportion of the number of people displayed at the end of treatment, 2 weeks after the end of exercise, and 6 weeks after the end of exercise showed a downward trend in both the rehabilitation group and the control group. The reason may be that all subjects stopped core strength training and electric traction therapy after the end of treatment. At the same time, all subjects must participate in training according to the training plan. Training cannot be stopped.

## 5. Conclusion

Chronic low back pain is a common disease of aerobics athletes, and it brings a lot of problems to aerobics athletes. To this end, a study on the effect of core strength training on aerobics athletes' chronic low back pain is presented. This article conducts research by setting up control experiments. There are experimental groups and control groups. The experimental group uses core strength training treatment. The control group uses electric traction treatment. The ODI questionnaire scores of the two groups are used to evaluate the treatment effect.

This study found that after core strength training, the ODI questionnaire scores were significantly different from before treatment, indicating that core strength training has a significant effect in helping patients with chronic low back pain to restore waist function. Compare the effectiveness of the core strength training treatment group and the traction treatment group in the treatment of chronic low back pain. In the four periods of evaluating the treatment effect, the scores of the core strength training group were lower than traction treatment in the ODI questionnaire scores in each period.

In addition, this article believes that core strength training is active in terms of training lumbar and abdominal muscle function. On the one hand, it can relieve the severity of chronic low back pain. On the other hand, the training of the lower back muscles can improve the structure and functional ability of the lumbar spine, and can have a beneficial effect on the characteristics of tissues such as bones, ligaments, tendons, and have a certain preventive effect on the occurrence of lower back pain.

The disadvantage of this article is that it limits the scope of rehabilitation training and can be developed in other areas, such as cervical spondylitis, and so on.

## Figures and Tables

**Figure 1:** Analysis of the scores of four ODI questionnaires in the experimental group.

**Figure 2:** Analysis of four ODI questionnaire scores in the control group.

**Figure 3:** Analysis of the average score changes of ODI questionnaire in the two groups.

**Figure 4:** Analysis of comparison results of ODI questionnaire scores between two groups.

**Figure 5:** Analysis of the proportion of subjects in each group whose ODI questionnaire scores significantly decreased.

**Table 1:** Basic information of subjects (*M*±SD).

Group	Number	Age (years)	Height (cm)	Weight (kg)
Experience group	30	18.10 ± 9.89	163.98 ± 4.92	58.71 ± 4.6
Control group	30	17.80 ± 12.39	163.10 ± 4.78	54.33 ± 6.2

**Table 2:** Comparison of ODI questionnaire scores between the two groups before and after treatment (*M*±SD).

Group	Before treatment	At the end of treatment	*P*
Experience group	38.33 ± 2.60	17.67 ± 6.67	0.001
Control group	38.56 ± 2.88	23.89 ± 7.51	0.02

**Table 3:** Comparison of ODI questionnaire scores between the two groups before and 2 weeks after treatment (*M*±SD).

Group	Before treatment	2 weeks after treatment	*P*
Experience group	38.33 ± 2.60	18.29 ± 2.32	0.001
Control group	38.56 ± 2.88	24.57 ± 1.59	0.029

**Table 4:** Comparison of ODI questionnaire scores between the two groups before and 6 weeks after treatment (*M*±SD).

Group	Before treatment	6 weeks after treatment	*P*
Experience group	38.33 ± 2.60	17.43 ± 3.21	0.001
Control group	38.56 ± 2.88	25.43 ± 3.26	0.037

## Data Availability

The data that support the findings of this study are available from the corresponding author upon reasonable request.
